The article "Is Surgery for Congenital Heart Defects in Neonates, Infants, and Children More Challenging and Demanding Than Surgery for Acquired Heart Defects in Adults?" was published in 2025. Journal: Cureus.

# Is Surgery for Congenital Heart Defects in Neonates, Infants, and Children More Challenging and Demanding Than Surgery for Acquired Heart Defects in Adults?

**DOI:** 10.7759/cureus.79765

**Published:** 2025-02-27

**Authors:** Sachin Talwar, Vishal V Bhende, Mathangi Krishnakumar, Krutika Tandon, Purvi R Patel

**Affiliations:** 1 Cardiothoracic and Vascular Surgery, All India Institute of Medical Sciences, New Delhi, New Delhi, IND; 2 Pediatric Cardiac Surgery, Bhanubhai and Madhuben Patel Cardiac Centre, Shree Krishna Hospital, Bhaikaka University, Karamsad, IND; 3 Anesthesiology, St. John’s Medical College Hospital, Bengaluru, IND; 4 Pediatrics, Pramukhswami Medical College, Shree Krishna Hospital, Bhaikaka University, Karamsad, IND

**Keywords:** congenital heart defects, family-centered care, global health disparities, intraoperative management, pediatric cardiac surgery

## Abstract

Pediatric cardiac surgery is a highly challenging medical subspecialty requiring technical precision, adaptability, and extensive multidisciplinary support. Unlike adult cardiac surgery, which often addresses standardized acquired conditions, surgery for congenital heart disease (CHD) in neonates, infants, and children involves unique anatomical and physiological complexities. These patients often need individualized surgical plans, and many benefit from staged interventions to accommodate growth. The steep learning curve for pediatric cardiac surgeons, combined with limited exposure to rare forms of CHD, underscores the importance of mentoring and specialized training. The limited cardiovascular reserve of younger patients makes them susceptible to physiological fluctuations, necessitating precise intraoperative management. Postoperatively, pediatric patients with CHD require intensive monitoring in specialized units and long-term follow-up because of their vulnerability to complications and delayed neurological developments. This field also places considerable psychosocial and financial burdens on families, highlighting the need for comprehensive, family-centered care. Global disparities in access to specialized resources perpetuate inequities in patient outcomes. Addressing these challenges requires a multidisciplinary approach integrating surgical expertise, holistic family support, and policy initiatives to improve worldwide access to care. Such a strategy is essential for advancing outcomes and ensuring equitable treatment for pediatric patients with CHD everywhere.

## Editorial

Unique anatomical and physiological challenges

A key distinction between surgery for congenital heart disease (CHD) and adult cardiac surgery lies in the conditions in each patient group. Adult procedures typically address conditions such as coronary artery disease, valvular disorders, or myocardial infarction, which often follow a standardized anatomical pattern. In contrast, surgery for CHD in neonates, infants, and children spans a broad range of structural anomalies, often requiring multi-staged procedures and more invasive open-heart surgeries tailored to the patient’s specific condition.

The article "Is Surgery for Congenital Heart Defects in Neonates, Infants, and Children More Challenging and Demanding Than Surgery for Acquired Heart Defects in Adults?" was published in 2025. Journal: Cureus.

CHD encompasses structural heart irregularities involving defects in the walls, cardiac chambers with their septae, valves, or blood vessels. Common congenital defects include ventricular septal defects, atrial septal defects, tetralogy of Fallot, and hypoplastic left heart syndrome (in neonates). Each defect differs in anatomical presentation and physiological impact, and many lead to chronic hypoxia that can adversely affect organ development. Surgeons frequently perform staged interventions to accommodate a child’s growth, improving long-term outcomes [1,2].

Additionally, the smaller and more delicate cardiac structures of younger patients require a high degree of technical precision. Surgical instruments, monitoring devices, and heart-lung machines must be adapted to pediatric anatomy. For instance, hypoplastic left heart syndrome requires complex staged repairs from the neonatal period because the entire left side of the heart is underdeveloped. Surgeons must account for ongoing growth and cardiac maturation. Grown-up congenital heart disease (GUCH) patients pose separate challenges and warrant different protocols, but GUCH is beyond our scope because this editorial focuses on pediatric populations.

The learning curve in pediatric cardiac surgery

Mastering congenital cardiac procedures in children involves one of the steepest learning curves in surgical subspecialties [3]. Complex technical skills and an extensive knowledge of varied anomalies are crucial. According to recent insights by Dr. Bacha, these aspects require years of practice aided by experienced mentors [4]. Trainees must develop the dexterity to operate on small, fragile hearts and manage the limited cardiovascular reserve of infants.

Traditional surgical training programs often offer insufficient exposure to the range of CHD conditions found in childhood. Although streamlined training can expedite specialization, it may also limit exposure to rarer congenital conditions. Consequently, mentorship programs are critical to helping young surgeons transition from theoretical knowledge to practical expertise, especially for complex CHD that benefits from the insights of senior surgeons [4].

In many centers, surgeons perform both acquired and congenital procedures, which can dilute the specialized skill set needed for pediatric cardiac surgery. Resource-intensive programs focusing solely on pediatric cases are less common, especially in private institutions. Public hospitals may perform more cardiac surgeries but still lack the specialized personnel and equipment to provide dedicated pediatric services. In countries like India, where many children are born with CHD [5], bridging the gap between initial diagnosis, referral to specialized centers, and achieving predictable surgical outcomes remains a significant challenge. Additionally, convincing parents to opt for surgery can be difficult, particularly in regions with high fertility rates, where factors such as financial constraints, cultural beliefs, and the perceived burden of multiple children influence decision-making.

The article "Is Surgery for Congenital Heart Defects in Neonates, Infants, and Children More Challenging and Demanding Than Surgery for Acquired Heart Defects in Adults?" was published in 2025. Journal: Cureus.

Intraoperative demands and patient stability

Physiological limitations in infants and children with CHD make intraoperative management complex. Younger patients have minimal cardiovascular reserves, leaving them susceptible to hemodynamic fluctuations, oxygen deprivation, and rapid metabolic shifts. Even minor oxygenation or blood pressure deviations can lead to critical complications, highlighting the need for close teamwork among surgeons, anesthesiologists, and perfusionists.

One study underscored the vital role of specialized anesthetic management in pediatric patients undergoing surgery for CHD, emphasizing continuous monitoring and adjustments to prevent instability [6]. Anesthesiologists often employ advanced techniques, such as near-infrared spectroscopy, to ensure adequate perfusion of the brain and other organs [7]. However such advanced monitoring is not commonly available even in top institutions. Balancing physiological stability requires experience, coordination, and swift intervention when needed.

Equipment and technology must also be tailored to pediatric patients. Miniaturized heart-lung machines, disposable oxygenators, and miniaturized coated tubing and circuits reduce the inflammatory response associated with cardiopulmonary bypass (CPB). The conduct of CPB flow rates, hypothermia levels, and circulatory arrest modified ultrafiltration differs significantly in children, whose vulnerability elevates the stakes for pediatric cardiac teams.

Postoperative care and intensive monitoring

Children with CHD need intensive monitoring and frequent follow-up after surgery. They are more prone to infections, arrhythmias, and respiratory complications than adults with acquired heart disease, requiring specialized pediatric intensive care units (PICUs) for continuous surveillance and rapid intervention. As these patients grow, new complications can arise, including bleeding, postoperative low cardiac output, and extended PICU stays. For example, older children with tetralogy of Fallot may need prolonged intensive care unit care due to myocardial hypertrophy, stiffness, and hypoxic cardiomyopathy stemming from longstanding cyanosis [8].

The article "Is Surgery for Congenital Heart Defects in Neonates, Infants, and Children More Challenging and Demanding Than Surgery for Acquired Heart Defects in Adults?" was published in 2025. Journal: Cureus.

Unlike adults, whose recovery tends to be more predictable, pediatric patients with CHD often face long-term follow-up and potential reoperations. PICUs are key in optimizing outcomes by closely monitoring and promptly managing unique pediatric complications [7,9]. However, global disparities persist. Specialized facilities and equipment are scarce in lower-resource regions, directly affecting postoperative care and long-term prognosis [10,11].

Family and psychosocial impact

Beyond technical challenges, pediatric cardiac surgery significantly affects families. Parents managing their child’s long-term care, including potential reoperations and intensive home care, often endure considerable emotional and logistical stress. Research shows that family-centered care, which incorporates psychological and social support, is crucial in addressing the complexities of pediatric cardiac surgery [12]. A multidisciplinary team, including social workers, psychologists, and other specialists, can help alleviate the burden faced by these families.

Because parents and caregivers serve as their children’s main advocates, family dynamics can become strained, especially when repeated hospital visits or additional surgeries are required. Balancing employment demands, other children’s needs, and financial constraints can be overwhelming. In many low-income countries, delays in treatment due to economic, cultural, or logistical factors can reduce the likelihood of timely surgery, increasing the risk of complications such as irreversible pulmonary artery hypertension. Furthermore, the lack of early intervention can lead to the progression of congenital heart defects into GUCH, necessitating complex management strategies and increasing the burden on healthcare systems. Limited awareness of favorable surgical outcomes also contributes to parents opting for more children rather than pursuing early intervention for the affected child [13].

For individuals with CHD, social acceptance may also be an issue, often complicating marriage, pregnancy, and employment opportunities. A medically and socially supportive environment helps mitigate these long-term psychosocial challenges.

Ethical and economic challenges

The ethical and financial dimensions of managing CHD in neonates, infants, and children add to the complexity. Severe cases have multiple comorbidities that often require lifelong care, resulting in significant medical expenses, particularly in resource-limited settings where specialized pediatric facilities may be inaccessible. To receive advanced cardiac services, families in certain areas must travel long distances or even cross national borders [14]. These burdens reveal the pressing need for policies that increase access to and affordability of specialized care.

The article "Is Surgery for Congenital Heart Defects in Neonates, Infants, and Children More Challenging and Demanding Than Surgery for Acquired Heart Defects in Adults?" was published in 2025. Journal: Cureus.

Ethical considerations further complicate decision-making. Providers and families must weigh surgical benefits against short- and long-term risks. Children with multiple or severe defects may face repeated surgeries and uncertain prognoses, challenging everyone involved to carefully evaluate the child’s future quality of life and the broader impact on the family [15].

Global disparities in access and resources

Inequitable access to pediatric cardiac care in infancy and childhood remains a major global health concern. Unlike adult cardiac care, which is often widely available, neonatal and pediatric procedures demand unique expertise and specialized equipment. Regions with limited resources frequently lack pediatric cardiologists, cardiac surgeons, and dedicated care units, resulting in avoidable disparities. Recent research highlighted the need for international collaboration and training initiatives to address these imbalances [16]. Sustained investments in education, infrastructure, and telemedicine are critical to improving outcomes in areas lacking advanced pediatric services (Figures 1, 2).

**Figure 1:** Comparative depiction of factors involved in adult and infant cardiac surgery. GUCH: grown-up congenital heart disease Image credits: Dr. Vishal V. Bhende and Dr. Mathangi Krishnakumar.

**Figure 2:** Pediatric cardiac surgery requires a comprehensive approach combining surgical skill, family support, and policies to improve global access to care than adult cardiac surgery. Image credits: Dr. Vishal V. Bhende and Dr. Mathangi Krishnakumar.

Conclusions

Surgery for CHD in neonates, infants, and children poses unique challenges beyond those encountered in adult cardiac procedures. The complexity of congenital heart defects, the requirement for growth-sensitive interventions, and the need for prolonged postoperative care underscore the specialized character of this field. Addressing these needs requires advanced technical skills, a holistic, family-centered approach, and a commitment to reducing global health disparities. By allocating appropriate training, resources, and policy support, the medical community can ensure that all pediatric patients with CHD receive the highest standard of care, regardless of geographic or socioeconomic limitations.
